The article "Correlation between Sputum Bacterial Culture Positive Rate and Drug Sensitivity Test Results and Disease Severity inInpatients and Its Clinical Significance: A SystematicReview and Meta-Analysis" was retracted in 2023. Reasons: unreliable results or conclusions; lack of ethics approval or compliance; concerns about the data; concerns about the peer review.

# Correlation between Sputum Bacterial Culture Positive Rate and Drug Sensitivity Test Results and Disease Severity inInpatients and Its Clinical Significance: A SystematicReview and Meta-Analysis

**DOI:** 10.1155/2022/5102100

**Published:** 2022-07-14

**Authors:** Wenjing Zhou, Jing Li

**Affiliations:** Department of Laboratroy Lianyungang TCM Hospital Affiliated to Nanjing University of Chinese Medicine, Lianyungang, Jiangsu 222004, China

## Abstract

**Objective:**

To systematically evaluate the correlation between the positive rate of sputum bacterial culture and the results of drug sensitivity test and the severity of the disease and its clinical significance, so as to provide evidence-based medicine for clinical application.

**Methods:**

PubMed, Embase, ScienceDirect, Cochrane Library, China Knowledge Network Database (CNKI), China VIP Database, Wanfang Database, and China Biomedical Literature Database (CBM) online database were used. The retrieval time limit was from the establishment of the database to the present. Data for all included studies were extracted by two independent researchers, and the risk of bias for the quality of each included study was assessed by the Cochrane Handbook 5.1.0 criteria. RevMan5.4 statistical software was used to analyze the collected data by meta.

**Results:**

In the end, 6 RCT articles were included. Overall, 613 samples were included in 6 RCT studies. The correlation between the positive rate of sputum bacterial culture in inpatients and the severity of the disease was meta-analyzed. The heterogeneity test results showed that Chi2 = 177.20, df = 3, *P* < 0.00001, and I^2^ = 98%, indicating that there was obvious heterogeneity among the included research data. It was considered that there was a correlation between the positive rate of sputum bacterial culture and the severity of the disease. The correlation between the results of the drug sensitivity test of inpatients and the severity of the disease was evaluated. The results of the heterogeneity test showed that Chi2 = 0.00, df = 1, *P* = 1 > 0.05, and I^2^ = 0%, indicating that there was no heterogeneity among the included research data. In addition, the combined effect of WMD was analyzed by the fixed effect model. The combined effect dose WMD test was *Z* = 6.58 (*P* < 0.00001). It was considered that there was a correlation between the results of the drug sensitivity test and the severity of the disease.

**Conclusion:**

There is a correlation between positive sputum culture and drug sensitivity test results and the severity of the disease in hospitalized patients. In clinical practice, for hospitalized patients, the positive sputum bacterial culture rate and drug sensitivity test results can be used to guide the appropriate use of antibiotics. Due to the low input from the literature, more studies with higher methodological quality and longer follow-up are needed for further validation.

## 1. Introduction

Pulmonary infection is a common respiratory disease. Influenza and pneumonia were combined as the eighth leading cause of death in the United States in 2011, according to the Centers for Disease Control and Prevention [1]. There are many kinds of pathogens that cause pulmonary infection, including bacteria, fungi, viruses, atypical pathogens, and parasites. Due to the widespread use of a variety of antimicrobials, the pathogen spectrum of pulmonary infection is diversified. According to relevant reports [2], the mortality rate of hospitalized pneumonia patients is 11.7%. The mortality rate of pneumonia patients in the pencil ICU is as high as 45% [3]. Without timely anti-infective treatment, it is easy to develop into cause systemic inflammatory response syndrome and then involve other organs, even lead to death of patients [4]. If antibiotics are abused, it will lead to an increase in the number of drug-resistant strains; if only empirical use of antibiotics, it is difficult to control infection, so it is necessary to select appropriate antibiotics according to the results of drug sensitivity. The selection methods of antibiotics for pulmonary infection include empirical selection and etiological diagnosis. Empirical drug selection is based on clinical data, previous pathogenic diagnosis, and experience in anti-infective treatment. Selection of anti-infective drugs that may be sensitive to anti-infective therapy was done. Etiological diagnostic drug selection refers to the method of selecting sensitive antibiotics for anti-infective treatment according to the results of the microbial culture and drug sensitivity test. When selecting drugs, the drug sensitivity test shows that they are sensitive to many kinds of antibiotics at the same time and then choose antibiotics with high sensitivity, narrow antibacterial spectrum, and low toxicity [5]. At present, some infection indexes such as C-reactive protein and procalcitonin are often used to diagnose pulmonary infection, but these indexes are lack of specificity. Bacteriological examination as a pathogen type of infectious disease is easy to be disturbed by many factors, so it is difficult to provide gold standard for disease diagnosis and treatment and its clinical application significance is low [6].

When bacterial infection occurs in human lungs or bronchi, the amount of sputum increases significantly. Sputum bacterial culture is performed by collecting the patient's sputum as a sample and growing the sample in a culture medium to observe the growth of bacteria. The identification of bacteria that have grown can identify the pathogenic bacteria in sputum, such as pneumococci, *Moraxella catarrhalis,* and *Klebsiella pneumoniae* [7]. It is helpful to the diagnosis and treatment of lower respiratory tract infectious diseases. In addition, the TB sputum culture cycle is long, usually taking half a month to a month, and it takes 2 months to get results for a complete dosing [8]. The pathogenic information of lung and bronchial lesions can be obtained through sputum culture, and then targeted intervention and treatment. The pharynx, larynx, and tonsils belong to the upper respiratory tract, and their diseases can also be obtained by expecting sputum culture to obtain pathogenic information. Based on the results of sputum culture, sensitive antibiotics can be selected. The drug sensitivity test is the abbreviation of the drug sensitivity test. The method is to take samples containing pathogenic bacteria from the infection site of the patient and inoculate them on a certain culture medium. At the same time, stick the paper with antibiotics on the surface of the culture medium and then observe the culture results. It is suitable to understand the sensitivity of pathogenic microorganisms to various antibiotics, so as to guide the rational selection of antibiotics in clinic. If a pathogen needs a small dose of antibiotics to inhibit and kill it, we say that the pathogen is sensitive to the antibiotic [9]. If a pathogenic bacterium needs a large dose of antibiotics to inhibit and kill it, we call it insensitive or resistant to this kind of antibiotics. If the pathogenic bacteria are sensitive to antibiotics, the larger the bacteriostatic circle is, and if the pathogenic bacteria are not sensitive to antibiotics, the smaller the bacteriostatic zone is. The size of the bacteriostatic zone is proportional to whether it is sensitive or not. The drug sensitivity test can guide the rational use of drugs [10]. Based on this, this study systematically evaluated the correlation between the positive rate of sputum bacterial culture and the results of the drug sensitivity test and the severity of the disease, as well as the clinical guiding significance, so as to provide evidence-based medicine for clinical use.

## 2. Research Contents and Methods

### 2.1. Sources and Retrieval Methods of Documents

The computer searched The Cochrane Library, Embase, PubMed, Web of Science, SinoMed, China Knowledge Network, Wanfang data knowledge Service platform, and VIP. The Chinese search words were “hospitalized patients, positive rate of sputum bacterial culture, results of drug sensitivity test, severity of disease, correlation, and clinical guiding significance.” The search time limit was to build each database to 2022–4.

### 2.2. Inclusion and Exclusion Criteria of Literature

#### 2.2.1. Literature Inclusion Criteria

(1) Research type: the randomized controlled trials (RCTs) were included on the correlation between sputum bacterial culture positive rate and drug sensitivity test results and disease severity in all inpatients in China. The language was limited to Chinese. (2) Participants: patients with positive rate of sputum bacterial culture were tested for drug sensitivity.

#### 2.2.2. Document Exclusion Criteria

(1) It was not a randomized controlled study. (2) The data report was incomplete and the data cannot be used. (3) Repeated the research content and the latest research. (4) The full text cannot be obtained.

### 2.3. Quality Evaluation and Data Extraction

1. Data for all included studies were extracted by two independent researchers, and the risk of bias for the quality of each included study was assessed by the Cochrane Handbook 5.1.0 criteria. The differences were resolved through discussion or asked the third researcher to negotiate and decide. The extracted data included the first author, year of publication, group, number of cases, age, prognosis index, and so on. The modified Jadad scale was used to evaluate the quality of the study, including the generation of random sequence (appropriate 2, unclear 1, and inappropriate 0), allocation concealment (appropriate 2, unclear 1, and inappropriate 0), blind (implementation 2, unclear 1, and unimplemented 0), and withdrawal and loss of follow-up (description 1 and undescribed 0). 0–3 was classified as low-quality research and 4–7 as high-quality research.
2. Data extraction: the extracted data were transformed as follows and then the data were analyzed by meta with RevMan5.0 software. The conversion formula is as follows [11]:

(1) $$\begin{array}{c} \text{Fisher's}Z:Z=0.5*\text{ln}\left(\frac{\left(1+r\right)}{\left(1-r\right)}\right),\\ Vz=\frac{1}{\left(n-3\right)},\\ Sez=Vz\Lambda 0.5,\\ r=\frac{\left(e\Lambda 2z-1\right)}{\left(e\Lambda 2z+1\right)}. \end{array}$$

### 2.4. Outcome Indicators

All the studies included were sputum bacterial culture positive rate and drug sensitivity test results to evaluate the severity of inpatients. The correlation between sputum bacterial culture positive rate and drug sensitivity test results to evaluate the severity of inpatients was expressed by Pearson correlation coefficient *r* value, so the Pearson correlation coefficient *r* value was used as the comprehensive outcome index. A negative value of *r* indicated a positive correlation between the positive rate of sputum bacterial culture and the results of the drug sensitivity test to evaluate the severity of hospitalized patients.

### 2.5. Statistical Processing

RevMan5 software was used for meta-analysis. Continuous variables were represented by standardized mean difference (SMD) and its 95%CI. If there was no statistical heterogeneity among the studies (*P* > 0.100, I2 <50%), the fixed effect model was used for analysis. Otherwise, the random effect model was used for analysis. If there was statistical heterogeneity, the sources of heterogeneity and subgroup were analyzed the factors that may lead to heterogeneity among the studies. If there is statistical heterogeneity but without clinical heterogeneity or statistically significant difference between the two groups, the random effect model was used for analysis. The sensitivity analysis was carried out by remerging the calculation after excluding the literature one by one. When the heterogeneity between the two groups was too large or unable to find the data source, descriptive analysis was used. Publication bias was analyzed by Egger's test. *P* < 0.05 means the difference is statistically significant.

## 3. Results and Analysis

### 3.1. The Literature Retrieval and the Basic Situation of Literature Inclusion

2133 articles were obtained by computer database search, and 432 articles were obtained after eliminating repeated studies. 56 articles were obtained from preliminary reading of titles and abstracts, irrelevant studies, reviews, case reports, and no control literature were excluded. 17 articles were initially included, and full text was carefully read. 11 articles with incomplete data and no main outcome indicators were excluded. Finally, 6 RCTs were included [12–17]. In total, 613 samples were analyzed by meta. The basic features included in the literature are shown in Table 1.

### 3.2. Evaluation of the Quality of the Methodology Included in the Literature

Six RCT literature studies were included to report the baseline of patients, and the included six studies all gave detailed intervention measures and follow-up time. RCT did not describe in detail the number and reasons of blindness and loss of follow-up or withdrawal. Risk bias is shown in Figure 1 and 2.

### 3.3. Results of Meta-Analysis

#### 3.3.1. Meta-Analysis of Fisher's *Z* Intermediate Conversion Value

Due to the large number of data, this paper only showed positive results.

#### 3.3.2. Correlation between the Positive Rate of Sputum Bacterial Culture and the Severity of the Disease

A total of 613 samples were included in 6 RCT studies. The correlation between the positive rate of sputum bacterial culture and the severity of the disease was analyzed by meta. The heterogeneity test results showed that Chi2 = 177.20, df = 3, *P* < 0.00001, and I^2^ = 98%, indicating that there was obvious heterogeneity among the included research data. It was considered that there was a correlation between the positive rate of sputum bacterial culture and the severity of the disease. The results are shown in Figure 3.

#### 3.3.3. Correlation between the Results of Drug Sensitivity Test and the Severity of the Disease

Six RCT studies were included with 613 samples. The correlation between the results of the drug sensitivity test and the severity of the disease in inpatients were assessed. The heterogeneity test results showed that Chi2 = 0.00, df = 1, *P* = 1 > 0.05, and I^2^ = 0%, indicating that there was no heterogeneity among the included research data, and the combined effect WMD was analyzed by the fixed effect model. The combined effect dose WMD test was *Z* = 6.58(*P* < 0.00001). It was considered that there was a correlation between the results of the drug sensitivity test and the severity of the disease. The results are shown in Figure 4.

## 4. Discussion

Nosocomial infections include infections that occur during hospitalization and acquired in the hospital but after discharge [18]. Nosocomial infections mainly include pneumonia, urinary tract infection, and hematogenous infection [19], which mostly occur in patients with mechanical ventilation, urinary catheterization, intravenous catheterization, and long-term use of antibiotics [20]. The common pathogens are *Klebsiella pneumoniae*, *Acinetobacter baumannii*, *Escherichia coli*, *Pseudomonas aeruginosa*, and *Staphylococcus aureus* [21]. Hospital-acquired infection is one of the main causes of death of critically ill patients [22]. The main cause of hospital-acquired infection is that the pathogenic bacteria develop drug resistance due to long-term or large-scale antibiotic treatment during hospitalization. Therefore, clinicians need to be familiar with and master the characteristics of hospital-acquired infection in actual work. This helps reduce the incidence of infection in patients. The current study showed that the main pathogens of hospital-acquired infection were Gram-negative bacteria dominated by *Acinetobacter baumannii*, *Pseudomonas aeruginosa*, *Klebsiella pneumoniae*, and *Escherichia coli*, Gram-positive bacteria dominated by *Staphylococcus aureus*, and fungi dominated by *Candida* [23]. The drug resistance of pathogens of hospital-acquired infection is suitable for the delayed use of antibiotics, which can not only increase the mortality of patients but also increase the drug resistance of bacteria in hospital [24]. Charles-Edouard Luyt et al. mentioned that 30% of the antibiotics used by hospitalized patients are unnecessary for patients and are not the most preferred antibiotics for the pathogen [25]. The long-term use of these antibiotics may lead to the emergence of bacterial resistance. To a certain extent, the distribution of bacteria is different from that in the general ward and the types of drug resistance of pathogens are wider than those in the general ward. Ramesh Venkataraman et al. analyzed the isolated strains of each flora collected, and in terms of the proportion of multiple drug-resistant bacteria [26]. The proportion of immobile bacteria, *Klebsiella*, *Escherichia coli*, *Pseudomonas*, and staphylococci was 87.5%, 75.5%, 61.9%, 58.9%, and 2.4%, respectively. Among Gram-negative bacteria, extended-spectrum *β*-lactamase-producing strains accounted for 34%, including *Klebsiella* (41.1%), *Escherichia coli* (26.4%), and *Pseudomonas* (23.5%). Carbapenem antibiotics are used as the first-line treatment of extended-spectrum *β*-lactamase-producing *Klebsiella pneumoniae* with the rapid increase of carbapenem-resistant strains, and the choice of antibiotic therapy is very limited [27]. Wirlaine Glauce Maciel et al. have believed that the production of metallo-*β*-lactamases is one of the important reasons for the resistance of *Pseudomonas aeruginosa* to *β*-lactam antibiotics including carbapenem antibiotics [28]. In their study, drug sensitivity tests showed that polymyxin B and colistin could be used as treatment options. The study of Voichița Lăzureanu et al. showed that the resistance rate of *Acinetobacter baumannii* to carbapenem antibiotics increased gradually [29]. Colistin was the only drug that maintained low resistance to *Acinetobacter baumannii* among the antibiotics used in this study. Ainihayati Noordin et al.'s research showed that 34% of methicillin-resistant *Staphylococcus aureus* (MRSA) was resistant to ciprofloxacin, ERY, and gentamicin, but sensitive to vancomycin and teicoplanin [30]. These reports suggest the prevalence of multi-drug-resistant bacteria, only a few advanced antibiotics maintain a low resistance rate, and some antibiotics cannot be used in some cases because of their side effects, resulting in more limited use of antibiotics.

Pulmonary infection can be life-threatening, especially for patients with low immune function and potential pulmonary dysfunction, such as cystic fibrosis and chronic obstructive pulmonary disease. According to the World Health Organization, lung infection was the leading cause of death in 2012. Eradicating lower respiratory tract infection is an arduous task [31]. Long-term use of antibiotics can easily lead to bacterial drug resistance. In view of bacterial drug resistance, if we do not selectively select sensitive antibiotics for pathogens, it will not only increase the economic burden but also delay the disease. Therefore, the etiological diagnosis of pulmonary infection is particularly important. The quality of sputum samples has a great influence on the diagnosis of sputum culture. Specimens from the lower respiratory tract may be contaminated by upper respiratory secretions during collection, and some poorly collected specimens may be composed entirely of upper respiratory secretions [32–35]. Either way, it can lead to the wrong conclusion that an organism that settles in the upper airway is causing pneumonia. Therefore, the standard practice of the diagnostic laboratory is to use indicators to evaluate the quality of sputum samples, which indicate that sputum samples are obtained from the lower respiratory tract. This includes evaluating the number of squamous epithelial cells (Secs) and polymorphonuclear cells (Pmns) in Gram staining smears [36]. Infection is a common complication of inpatients, and it may lead to prolonged hospitalization and high medical costs and even lead to death, so the prevention of infection is particularly important. Preventive measures mainly include the following: (1) strict central venous catheterization nursing. After 15 days of catheterization, the incidence of hematogenous infection increased sharply [37]. Therefore, regular removal and replacement of tubes should be taken into consideration. (2) Limit the application of acid inhibitors. Acid inhibitors can increase the incidence of delayed septicemia with the extension of time. The incidence will gradually increase, especially Gram-negative bacilli and fungal septicemia [38]. (3) Oral care and withdrawal as soon as possible. Sean van Diepen et al. have believed that raising the head of the bed, oral care with chlorhexidine and withdrawing the machine as soon as possible can reduce ventilator-associated pneumonia [36]. (4) Clean environment and hand hygiene. Patti et al. believed that a clean environment can reduce the spread of pathogens [39]. The hands of health care workers in the intensive care unit can also pollute the indoor environment after being contaminated, including the head of the patient's bed and sphygmomanometer cuff, which can also increase the risk of infection. (5) Limit the use of antibiotics. The study has shown that contact isolation, hand hygiene, and antibiotic control can be used as basic preventive measures for methicillin-resistant *Staphylococcus aureus* and multi-drug-resistant *Acinetobacter baumannii* infection [40–42]. Some scholars feel that communication and continuing education can reduce central venous catheter-related blood flow infection [43]. Typically, hospitalized patients are critically ill, in poor baseline condition, and the pathogens are mostly multi-drug-resistant bacteria. The choice of antibiotics available is very limited, and treatment is difficult, factors that can lead to a poor prognosis or even death.

Finally, we included 6 RCT articles. A total of 613 samples were analyzed by meta. The correlation between the positive rate of sputum bacterial culture and the severity of the disease was analyzed by meta. The results of the heterogeneity test showed that Chi2 = 177.20, df = 3, *P* < 0.00001, and I^2^ = 98%, indicating that there was obvious heterogeneity among the included research data. In addition, it was considered that there was a correlation between the positive rate of sputum bacterial culture and the severity of the disease. Through the inclusion of 6 RCT studies, the correlation between the results of the drug sensitivity test of inpatients and the severity of the disease was analyzed by meta. The results of the heterogeneity test showed that Chi2 = 0.00, df = 1, *P* = 1 > 0.05, and I^2^ = 0%, indicating that there was no heterogeneity among the included research data, and the combined effect of WMD was analyzed by the fixed effect model. The combined effect dose WMD test was *Z* = 6.58 (*P* < 0.00001). It can be considered that there was a correlation between the results of the drug sensitivity test and the severity of the disease. Due to the status of inpatients and the application of invasive measures, there is a high incidence of infection. This prolongs hospital stays and even aggravates the condition, leading to death [44–46]. Generally, culture drug sensitivity tests for pathogenic bacteria take a long time and require empirical treatment by the physician. The resistant and heterogeneous nature of the infecting bacteria, as well as the underlying illness of the patient, make it impossible for the patient to use some antibiotics, which makes it very difficult for doctors to use empirical drugs. Therefore, the sputum culture test is used to determine whether patients are infected with bacteria. Combined with the results of the drug sensitivity test, medication for patients can achieve rational use of drugs and achieve the purpose of treating diseases [47].

In conclusion, there is a certain correlation between the sputum bacterial culture positive rate and drug sensitivity test results of inpatients and the severity of the disease. Based on the results of sputum culture, sensitive antibiotics can be selected for hospitalized patients. Due to less literature input, more studies and follow-up with higher methodological quality are needed for further verification.

## Figures and Tables

**Figure 1:** Risk of bias assessment of included studies.

**Figure 2:** Summary chart of risk bias of included studies.

**Figure 3:** Forest plot of the positive rate of sputum bacterial culture and the severity of the disease.

**Figure 4:** Forest plot of drug sensitivity test and the severity of the disease.

**Table 1:** Basic characteristics of the literature.

Include the literature	Year of publication	*N*	Age	Average age	Disease type	Correlation coefficient between the positive rate of sputum bacterial culture and the severity of disease	Correlation coefficient between the results of drug sensitivity test and the severity of the disease	Conclusion
Fan Xin	2019	53	24–77	53.47 ± 6.38	Pneumonia	*r* = −0.495	-	Most of the patients with acute exacerbation of bronchiectasis were positive for sputum culture, suggesting that there was a certain correlation between the severity of the disease and the positive results of sputum culture.
Tian Yu	2015	60	33–68	50.4 ± 7.2	Chronic obstructive pulmonary disease	*r* = −0.673	-	Sputum culture was positive, indicating that the patient had bacterial infection, and AECOPD was related to the severity of bacterial infection.
Zhao Mingli	2013	100	68–89	78.38 ± 5.87	Chronic obstructive pulmonary disease	*r* = −0.839	-	Pulmonary fungal infection, especially *Aspergillus* infection, may be one of the causes of persistent wheezing in patients with chronic obstructive pulmonary disease.
Zhang Yaodong	2012	96	25–56	36.93 ± 4.53	Pneumonia	-	*r* = 0.732	The drug resistance rate of most bacteria is positively correlated with the frequency of antibiotics. According to the disease severity of inpatients, the monitoring of bacterial drug resistance and the management of clinical application of antibiotics should be strengthened.
Zhong Jiao	2011	104	33–84	56.39 ± 4.34	Pneumonia	-	*r* = 0.811	The drug resistance of bacteria is related to the severity of the disease in inpatients, suggesting that the clinical use of antibiotics should be standardized to reduce the production of drug-resistant bacteria.
Peng Min	2008	200	6–34	15.39 ± 2.44	Acute attack of bronchial asthma	*r* = 0.133	-	The main inducing factors of asthma attack were upper respiratory tract infection, followed by dust mites, house dust, and pollen. Lower respiratory tract infection is relatively rare, and the positive rate of sputum culture is low, which is not the main inducing factor of asthma attack.

## Data Availability

No data were used to support this study.
